# HNF-4α inhibits hepatocellular carcinoma cell proliferation through mir-122-adam17 pathway

This article has been retracted.

**DOI:** 10.1371/journal.pone.0230450

**Published:** 2020-03-25

**Authors:** Guang Yang, Min Zhang, Yawei Zhao, Yue Pan, Mujie Kan, Jing Li, Kan He, Xuewen Zhang

**Affiliations:** 1 Department of Hepatobiliary and Pancreatic Surgery, The Second Affiliated Hospital of Jilin University, Changchun, Jilin, China; 2 Department of Pharmacology, College of Basic Medical Sciences, Jilin University, Changchun, China; 3 Department of Biochemistry, College of Basic Medical Sciences, Jilin University, Changchun, China; Chung Shan Medical University, TAIWAN

## Abstract

Hepatocellular carcinoma (HCC) is one of the most common human cancers, its prevalence and severity need us to discover novel early diagnostic biomarkers and new therapeutic strategies. MicroRNA-122 is the most abundant microRNA in the liver, and acts as a tumor suppressor and represses HCC development. In our study we showed that HNF-4α and MiR-122 were down-regulated significantly in hepatocellular carcinoma. Over-expression of HNF-4α inhibit hepatocellular carcinoma cells proliferation. And miR-122 is one of the downstream effector of HNF-4α. Up-regulated miR-122 inhibited hepatocellular carcinoma cells proliferation through regulating ADAM17. Collectively, our results suggested that HNF-4α could inhibit hepatocellular carcinoma proliferation with miR-122 being a downstream target of it. And miR-122 would inhibit hepatocellular carcinoma proliferation by regulating ADAM17 signal pathway.

## Introduction

The incidence and mortality of hepatocellular carcinoma (HCC) is both very high among human cancers, affecting a lot of people each year worldwide. Approximately 782,500 newly diagnosed cases were found and 745,500 patients died of liver cancer worldwide in 2012, among which nearly half of the total number of cases and deaths were in China [1]. It is the 2^nd^ leading cause of cancer-related death in males and the third in females, with a total mortality rate of 26.3 per 100,000 in China[2]. Despite of the success in the traditional therapies including surgery or transcatheter arterial chemoembolization, the recurrence rate in HCC patients is still high due to the intrahepatic metastasis and local invasion. Given this context, there is an urgent need to discover novel early diagnostic biomarkers and new therapeutic strategies for HCC.

Although various genetic and epigenetic changes that lead to HCC have been revealed, the underlying molecular mechanisms for liver cancer are not fully elucidated. MicorRNAs (miRNAs), discovered by Ambros and colleagues in 1993[3], are small noncoding RNAs. The length of miRNAs is 18–24 nucleotides. Through binding to the 3’-untranslated region (3’-UTR) of their target mRNAs, they can inhibit the expression of the target genes by the cleavage or repressing the translation of the target mRNAs [4]. Recent research highlighted the role of dysregulated microRNAs in HCC. MicroRNA-122, a liver specific miRNA, accounts for 70% of the total liver miRNA population, which is significantly down-regulated in most hepatocellular carcinomas (HCCs) but its role in tumorigenesis remains poorly understood. Tsai demonstrated that deletion of the gene encoding miR-122 in mice leads to the development of steatohepatitis, fibrosis and HCC[5]. MiR-122 acts as a tumor suppressor and represses hepatocellular carcinoma (HCC) development by binding to target genes involved in the process of angiogenesis, differentiation, proliferation, apoptosis and migration in HCC[6]. However, the effects of miR-122 in HCC have not been completely elucidated. Therefore, it is of great significance to further study the function and mechanism of miR-122 in HCC.

The expression of miR-122 is correlated with liver-enriched transcription factors (LETFs), such as hepatocyte nuclear factor (HNF1α, HNF3α, HNF3β, HNF4α, HNF6), and C/EBPα[7–9]. These LETFs are coordinately involved in the transcriptional regulation of miR-122 by binding to the miR-122 promoter as transcriptional activators. Li showed that HNF4α positively regulates miR122 expression in both Huh7 cells and the mouse liver, suggesting that HNF4α is a key regulator of miR-122 expression in the liver[8].

In this study we investigated the potential function of miR-122 in the development and progression of HCC. We firstly investigated whether HNF-4α and miR-122 could affect the hepatocarcinogenesis, then revealed the relationship between HNF-4α and miR-122 and investigated the molecular mechanisms of HNF-4α and miR-122 inhibiting hepatocellular carcinoma.

## Materials and methods

### Acquisition and preprocessing of microarray data

Firstly, we studied differentially expressed genes (DEGs) in hepatocellular carcinoma tissues and adjacent non-cancerous tissues of hepatocellular carcinoma patients at the mRNA level. We used hepatic carcinoma-associated dataset GSE84402 [10] in Gene Expression Omnibus (GEO) database (http://www.ncbi.nlm.nih.gov/geo). The GSE84402 dataset contained 14 human hepatocellular carcinoma tissues samples and 14 corresponding non-cancerous tissues samples of hepatocellular carcinoma patients. The samples were profiled using the chip-based platform GPL570. The preprocessed gene expression matrix of dataset GSE84402 was downloaded from the GEO database.

We also studied DEGs in hepatocellular carcinoma tissues and adjacent non-cancerous tissues at the microRNA level. we used hepatic carcinoma-associated dataset GSE54751 [11–13] in GEO database. The GSE54751 dataset contained 10 HCC tumor tissues samples and 10 adjacent non-tumor tissues samples of hepatocellular carcinoma patients. The samples were profiled using the chip-based platform GPL18262. The preprocessed gene expression matrix of dataset GSE54751 was downloaded from the GEO database.

Before analyzing DEGs, we filtered the probes without known gene symbols, and the probe-level expression profiles for the dataset were converted to gene-level expressions by using the collapseRows function to merge probes [14].

### Analysis of DEGs

Microarray data analysis was performed using R software and Bioconductor 3.3.2 (http://www.bioconductor.org/). We used R Limma package [15] to identify DEGs between hepatocellular carcinoma tissues and adjacent non-cancerous tissues samples of hepatocellular carcinoma patients. The fold change > 2 and P < 0.05 were regarded as the threshold of differential expression.

### Tissue samples

This study was approved by the Ethics Review Committees of China-Japan Union Hospital, Jilin University, and written informed consent was obtained from all patients. A total of 40 patients with HCC had undergone routine surgery at China-Japan Union Hospital, Jilin University. HCC samples and the matched pericarcinomatous tissues taken from these 40 patients were immediately frozen in liquid nitrogen and stored at -80°C or fixed in 10% formalin for paraffin embedding.

### Cell culture

The human liver cancer cell lines HepG2, Bel-7402, and Bel-7404 and the normal human hepatic embryo cell line HL-7702 were obtained from the Chinese Academy of Sciences (Shanghai, China). We conduct mycoplasma testing by PCR during culture routinely; no addition authentication was done by the authors. Cells were cultured in DMEM (GIBCO, Carlsbad, CA, USA) supplemented with 10% FBS (Beijing Dingguo Biological Technology Co., Ltd. Beijing, China), 100 U/ml penicillin, and 100 mg/ml streptomycin at 37°C in a humidified atmosphere of 95% air and 5% CO_2_.

### Cell transfection with miRNA

HepG2 cells were transfected with miR-122 mimic or negative control (NC) at 100 nM. miR-122 mimic (5′-CAAACACCAUUGUCACACUCCA-3′) and negative control (5′-CAGUACUUUUGUGUAGUACAA-3′) were purchased from RiboBio Co., Ltd., Guangzhou, China. FITC labelled NC was purchased and used to measure the transfection efficiency under fluorescence microscope. The transfection efficiency was approximately 90%.

### RNA extraction and quantitative real-time polymerase chain reaction

Total RNA and miR fractions were isolated from tissue samples and the HepG2, Bel-7402, Bel-7404 and HL-7702 cell lines using TRIzol reagent (Invitrogen, Carlsbad, CA, USA). RNA was reverse transcribed into cDNA using the TransScript First-Strand cDNA Synthesis SuperMix (TransScript) (Invitrogen), following the manufacturer’s instructions. MiRNA extraction was performed using the miRNA Extraction Kit (Tiangen, Beijing, China). Quantitative real-time polymerase chain reaction (qRT-PCR) was performed on the FastStart Universal STBR Green Master (ROX) (Roche, Basel, Switzerland). Primers for miR-122 3p and U6 were obtained from RiboBio (Guangzhou, China). The expression of miR-122 was normalized to that of U6 using the 2^-ΔΔct^ method.

### Cell viability assay

Cells were seeded in 96-well plates at 5 × 10^3^ cells per well and transfected with 100 nmol/L miR-122 mimic, 200 nmol/L miR-122 mimic or HNF-4α plasmid (Santa Cruz Co., Ltd Shanghai, China), and were further incubated for 24 h. Thereafter, cells were incubated in 0.1 mg/ml MTT (Sigma, St. Louis, MO, USA) at 37°C for 3 h and lysed in dimethyl sulfoxide at room temperature for 30 min. The absorbance in each well was measured at 490 nm using a microplate reader. Each experiment was performed in triplicate.

### Western blot analysis

Cells were collected and lysed in 0.1 ml cold RIPA lysis buffer containing 0.02% phenylmethanesulfonyl fluoride. The cell lysates were then centrifuged at 12,000 ×g for 30 min at 4°C. Protein concentrations were determined with the Bradford Protein Assay Kit (Beyotime Institute of Biotechnology, Beijing, China), using bovine serum albumin as the standard. The proteins were separated by SDS-polyacrylamide gel electrophoresis and transferred to polyvinylidene difluoride membranes. After nonspecifc binding sites had been blocked with 5% nonfat dry milk in PBS for 60 min, the transferred membranes were incubated overnight at 4°C with primary antibodies. Following repeated washes with Tris buffered saline with 0.1% Tween (TBST), the membranes were incubated with horseradish peroxidase (HRP)-conjugated mouse anti-rabbit secondary antibody or HRP-conjugated rabbit anti-mouse secondary antibody for 1.5 h at room temperature prior to additional washes with TBST. Detection of antibody binding was performed using the enhanced chemiluminescence kit. Equal loading was verified using antibodies against glyceraldehyde-3-phosphate dehydrogenase. All Western blot analyses were repeated 3 times. Quantification of the protein expression was analyzed by Quantity One software.

### Statistical analysis

All data were analyzed for statistical significance using GraphPad Prism software. Data were expressed as the mean ± standard deviation (SD). Statistical analysis was performed using nonpaired t-test for single comparisons or one-way analysis of variance for multiple comparisons, and a P < 0.05 was considered to be statistically significant.

## Results

### MiR-122 is down-regulated significantly in hepatocellular carcinoma tissues and cell lines

To investigate the expression level of miR-122 between clinical HCC and matched pericarcinomatous tissues from 40 HCC patients, the expression was measured by qRT-PCR. As showed in Fig 1A, the expression of miR-122 was significantly lower in HCC than that in the non-tumor liver samples. We further evaluated the expression of miR-122 in hepatocellular cell lines HepG2, Bel-7402 and Bel-7404, as well as in the normal human hepatocyte HL-7702 cell line. MiR-122 was down-regulated in all tested HCC cell lines compared with the HL-7702 cell line (Fig 1B). Besides, we used hepatic carcinoma-associated dataset GSE54751 (11–13) in GEO database to confirm the deregulation of miR-122 in hepatocellular carcinoma. In GSE54751 data set, including miR-122, a total of 5 differentially expressed genes between hepatocellular carcinoma tissues and adjacent non-cancerous tissues samples of hepatocellular carcinoma patients were found, among which 2 up-regulated genes (hsa-miR-17 and hsa-miR-106a) and 3 down-regulated genes (hsa-miR-122, hsa-miR-1274b and hsa-miR-223) were identified using fold change >2 and P<0.05 (Fig 1C and 1D).

**Fig 1:** MiR-122 expression in hepatocellular carcinoma (HCC) cell lines and tissues. **(A)** MiR-122 expression was examined by quantitative real-time polymerase chain reaction (qRT-PCR) in human HCC tissues and adjacent normal tissues (control group); **(B)** qRT-PCR analysis of miR-122 expression in normal liver cells (HL-7702, as control group) and three HCC cell lines (HepG2, Bel-7402 and Bel-7404). MiR-122 expression in each sample was normalized to that of U6, the internal control (*P < 0.05 vs. control group). **(C)** Volcano plot of the DEGs. DEGs were selected with P < 0.05 and fold change > 2. **(D)** DEGs can be effectively divided into hepatocellular carcinoma tissues and adjacent non-cancerous tissues groups. Up-regulated and down-regulated genes were represented by red and green, respectively.

### Up-regulated miR-122 inhibited hepatocellular carcinoma cells proliferation through regulating ADAM17

To explore the effect of miR-122 on hepatocellular carcinoma cells proliferation, miR-122 mimic (miR 122 (+)) was used to mimic up-regulation miR-122 in HepG2 cells following with MTT assay. As showed in Fig 2A, proliferation of HepG2 cells was significantly inhibited by miR-122 mimic. The expressions of several validated downstream signaling components of miR-122 were also detected after miR-122 mimic treatment in HepG2 cells. As shown in Fig 2B–2F, miR-122 mimic down-regulated ADAM17, EGFR, p-AKT but increased the cleaved Caspase 3.

**Fig 2:** Up-regulated miR 122 inhibited hepatocellular carcinoma cells proliferation through regulating ADAM17. **(A)** MTT assay of HepG2 cells transfected with miR-122 mimic for 24 h *in vitro*. **(B)** HNF-4α, ADAM17, EGFR, AKT, p-AKT, F-Caspase 3 and C-Caspase 3 protein expression in HepG2 cells transfected with miR-122 mimic at 200 nM. Relative quantification of western blot results ADAM17 **(C)**, EGFR **(D)**, p-AKT/AKT **(E)**, and cleaved caspase 3/caspase 3 **(F)** levels expressed relative to control. (*P < 0.05 vs. the control). CON: control; NC: negative control.

### Over-expression of HNF-4α inhibits hepatocellular carcinoma cells proliferation through regulating miR-122

To study whether HNF-4α regulates miR-122 in HCC, HNF-4α plasmid (HNF-4α (+)) was used to transfect HepG2 cells. As shown in Fig 3A and 3B, HNF-4α plasmid up-regulates the expression of miR-122, indicating that the expression of miR-122 is controlled by HNF-4α. Moreover, the expression of the proliferation related proteins ADAM17, EGFR, and p-AKT which are the downstream of miR122 were inhibited and Caspase 3 was activated (Fig 3C–3F). Similar with results above, activation of Caspase-3 was also observed after HNF-4α plasmid transfection in HepG2 cells (Fig 3G). Finally, proliferation of HepG2 was significantly inhibited by HNF-4α plasmid (Fig 3H).

**Fig 3:** Over-expressions of HNF-4α inhibit hepatocellular carcinoma cells proliferation through regulating miR-122. **(A)** HNF-4α, ADAM17, EGFR, AKT, p-AKT, F-Caspase 3 and C-Caspase 3 protein expression in HepG2 cells transfected with HNF-4α plasmid for 24 h. **(B)** qRT-PCR analysis of miR-122 expression in HepG2 cells transfected with HNF-4α plasmid for 24 h. Relative quantification of western blot results HNF-4α **(C)**, ADAM17 **(D)**, EGFR **(E)**, p-AKT/AKT **(F)**, and cleaved caspase 3/caspase 3 **(G)** levels expressed relative to control. **(H)** MTT assay of HepG2 cells transfected with HNF-4α plasmid for 24 h *in vitro*. (*P < 0.05 vs. the control). CON: control; NC: negative control.

### HNF-4α is down-regulated in hepatocellular carcinoma

Since we found that over-expression of HNF-4α inhibits hepatocellular carcinoma cells proliferation, we come back to explore the expression pattern of HNF-4α in hepatocellular carcinoma cell lines. Similar with the expression trend of miR-122 in HCC (Fig 1B), the protein expression of HNF-4α was significantly decreased in all three hepatocellular cell lines HepG2, Bel-7402 and Bel-7404, compared with normal human hepatocyte HL-7702 cell line (Fig 4A and 4B). Oppositely, the expression of downstream target gene of miR-122 was significantly higher in three hepatocellular cell lines (Fig 4A, 4C and 4D). Moreover, by using Limma package of R software, in GSE84402 data set, a total of 3603 differentially expressed gene between hepatocellular carcinoma tissues and adjacent non-cancerous tissues samples of hepatocellular carcinoma patients were analyzed, among which 2246 up-regulated genes and 1357 down-regulated genes were identified using fold change >2 and P<0.05 (Fig 4E and 4F). The 3603 differentially expressed genes of hepatocellular carcinoma were further analyzed by hierarchical clustering. The general gene expression patterns in the two groups were significantly different by TreeView (Fig 4G). These results confirmed that HNF-4α is down-regulated in hepatocellular carcinoma.

**Fig 4:** HNF-4α is down-regulated in hepatocellular carcinoma cell lines. **(A)** HNF-4α, ADAM17 and EGFR protein expression in normal liver cells (HL 7702, as control group) and three HCC cell lines (HepG2, Bel 7402 and Bel 7404). Relative quantification of HNF-4α **(B)**, ADAM17 **(C)**, and EGFR **(D)** levels expressed relative to control. (*P < 0.05 vs. the control). **(E)** Histogram plot of the DEGs. DEGs were selected with P < 0.05 and fold change > 2. **(F)** Volcano plot of the DEGs. DEGs were selected with P < 0.05 and fold change > 2. **(G)** DEGs can be effectively divided into hepatocellular carcinoma tissues and adjacent non-cancerous tissues groups. Up-regulated and down-regulated genes were represented by red and green, respectively.

## Discussion

The prevalence and severity of HCC are increasing worldwide, and the prognosis of HCC patients remains unsatisfactory due to the high rate of recurrence and metastasis. Therefore, improved therapeutic strategies for HCC patients are critical for the management of HCC. In our study, we investigated the potential function of miR-122 in the development and progression of HCC. The relationship between HNF-4α and miR-122 and the molecular mechanisms of HNF-4α and miR-122 in inhibiting hepatocellular carcinoma were revealed.

MiRNAs have recently emerged as new anticancer drugs because they exert antitumor properties in a wide range of tumor cell types, including HCC cells. The emerging role of dysregulated miRNAs in HCC has been shown in many studies. Therefore, a better understanding of the roles of miRNAs in the pathogenesis of malignancy may help in the search for more effective HCC therapies. A number of studies have revealed the miRNA profile of HCC. Many miRNAs are aberrantly expressed in HCC and function as oncogenes or tumor suppressors[16].

MiR-122 is the most frequently detected miRNA in liver[17] whose existance is also confirmed in blood and serum. It is shown that in non-alcoholic fatty-liver disease (NAFLD) and chronic hepatitis B or C, MiR-122 can be a biomarker indicating the existence of liver injury [18,19]. Decreased miR-122 levels have been associated with poor prognosis and metastasis of hepatocellular carcinomas, and several targets of miR-122 have been implicated in tumorigenesis, including ADAM10, cyclin G1, SRF, Wnt1 and IGF1R [20]. These data suggested that miR-122 acts as a tumor suppressor in the liver, but its role in tumorigenesis remains poorly understood.

Hepatocyte nuclear factors (HNF) play a critical role in development of the liver. They take part in the maintenance of hepatocyte differentiation and the expression of liver-specific genes, and also play important roles in liver tumorigenesis and progression of HCC. Natalia Lazarevich et.al. elucidated the role of liver transcription factors in HCC progression through the generation of a novel *in vivo* experimental model demonstrating that a low-invasive slow-growing transplantable differentiated mouse HCC (sgHCC) rapidly given rise to a highly invasive dedifferentiated fast-growing variant (fgHCC). They demonstrated the critical role of HNF4 in HCC progression towards a more aggressive phenotype[21].

In our results, the expression of HNF4α was decreased in the hepatocellular carcinoma cell lines, and miR122 expression was reduced in hepatocellular carcinoma tissues and cell lines compared with the normal liver tissue and liver cells. In our study, regarding to the normal hepatocyte cells we used were not adult hepatocyte cells but an established cell line of embryonic cells, the gene expression could differ from normal adult cells. And the over-expressed HNF-4α would inhibit HepG2 proliferation and promote the expression of miR122. Those results further confirmed that HNF4α is a key regulator of miR-122 expression in the liver and they play important roles in liver tumorigenesis and progression of HCC. So we proposed that loss of HNF4 expression was a critical event during HCC progression. And the decreased expression of miR122 might be one of the mechanisms of HCC.

ADAM17 is one target of miR-122 and is implicated in numerous human diseases including cancer, heart disease, diabetes, rheumatoid arthritis, kidney fibrosis, Alzheimer’s disease, and it is a promising target for future treatments. ADAM17 plays a critical role in development of liver tumorigenesis and progression in hepatocellular carcinomas [22]. Tsai found that silencing of ADAM17 resulted in a dramatic reduction of in vitro migration, invasion, in vivo tumorigenesis, and angiogenesis, which is similar to that which occurs with the restoration of miR-122[22]. In our results, ADAM17 expression was reduced in hepatocellular carcinoma cell lines compared with liver cells. And proteins EGFR, AKT, Caspase 3 which are associated with tumor growth were regulated by ADAM17 in our research. Consistently, we showed that transfection of the miR-122 mimic suppressed the proliferation of HepG2 cell lines. Over-expressed HNF-4α and the miR-122 mimic could reduce ADAM17 expression. ADAM17 is regulated by HNF-4α and miR-122.

In summary, this work showed that over-expressed HNF-4α could inhibit hepatocellular carcinoma proliferation. And miR-122 is one of the downstream effectors of HNF-4α. And miR-122 would inhibit hepatocellular carcinoma proliferation by regulating ADAM17 signal pathway.

## Supporting information

S1 Raw images (PDF)
